# LncRNA DQ786243 contributes to proliferation and metastasis of colorectal cancer both *in vitro* and *in vivo*

**DOI:** 10.1042/BSR20160048

**Published:** 2016-05-06

**Authors:** Longci Sun, Hanbing Xue, Chunhui Jiang, Hong Zhou, Lei Gu, Ye Liu, Chunjie Xu, Qing Xu

**Affiliations:** * Department of Gastrointestinal Surgery, Renji Hospital, School of Medicine, Shanghai Jiao Tong University, Shanghai 200127, China; † Department of Gastroenterology, Renji Hospital, School of Medicine, Shanghai Jiao Tong University, Shanghai 200127, China

**Keywords:** colorectal cancer (CRC), invasion, long non-coding ribonucleic acid (LncRNA), migration

## Abstract

Accumulating evidence demonstrates that long non-coding RNAs (LncRNAs) play important roles in regulating gene expression and are involved in various cancers, including colorectal cancer (CRC). However, LncRNA profiles in CRC remain largely unknown. The present study aims to find the key LncRNA associated with CRC and to study its biological functions in CRC progression. We focused on LncRNA DQ786243, one of LncRNAs which promoted development of CRC from the Gene Expression Omnibus (GEO) and validated using quantitative real-time PCR among about 20 paired CRC tissues. The effects of LncRNA DQ786243 were assessed by silencing the LncRNA *in vitro* and *in vivo*. Results showed that the expression level LncRNA DQ786243 was significantly higher in CRC tissues and cell lines. We also found LncRNA DQ786243 knockdown by RNA interference with siRNA significantly arrested the cell cycle in the G_2_/M-phase, promoted apoptosis and weaken the abilities of cell proliferation and invasion *in vitro*. Further investigation into the mechanisms responsible for the growth inhibitory effects by DQ786243 silencing revealed that its knockdown resulted in the induction of cell cycle arrest and apoptosis through certain cell cycle-related and apoptosis-related proteins. Finally, xenograft experiments confirmed that the growth of xenograft tumours formed by CRC cells was suppressed after silencing LncRNA DQ786243 expression. In conclusion, the present study suggests that LncRNA DQ786243 is an oncogene that promotes tumour progression and leads us to propose that LncRNAs may serve as key regulatory hubs in CRC progression.

## Abstract (precis)

This article aims to find the key long non-coding RNAs (LncRNAs) associated with colorectal cancer (CRC) and to study its biological functions in colorectal cancer progression. Our study has shown that upregulated LncRNA DQ786243 can regulate cell proliferation, cell cycle progression, cell apoptosis, migration, and invasion in CRC cells. Xenograft experiments confirmed that the growth of xenograft tumors formed by CRC cells was suppressed after silencing LncRNA DQ786243 expression. In conclusion, our study suggests that LncRNA DQ786243 is an oncogene that promotes tumor progression and leads us to propose that LncRNAs may serve as key regulatory hubs in CRC progression.

## INTRODUCTION

Colorectal cancer (CRC), which ranks the third in the cancer morbidity and the second in the cancer mortality, is the most prevalent malignant cancer in the world with annual new cases exceeding 1000000 [1]. Colorectal carcinogenesis is a multistep process including progressive disruption of epithelial cell proliferation, apoptosis, differentiation and survival mechanisms [2,3]. Due to the chemotherapy and radiation therapy, the incidence and mortality of CRC are decreased in recent years. But the 5-year survival rate of CRC patients remains relatively low. Therefore, it is important to find effective methods for early diagnosis and treatment of CRC.

Long non-coding RNA (LncRNA) is a type of RNA molecule with length of more than 200 bp and lacks an open reading frame of significant length and the capability of coding protein [4–7]. Unlike the smaller non-coding miRNAs, the functions of the majority of LncRNAs are not fully clear. However, with the improvement of technology and research in transcriptome profiles, some LncRNAs were reported to be abnormally expressed in various cancers and were associated with tumour cell proliferation, growth, apoptosis, invasion and metastasis [8–14]. When it comes to CRC, several LncRNAs played important role in CRC, such as HOTAIR, HULC and H19. For example, HOTAIR is a cancer-related LncRNA that can regulate polycomb-dependent chromatin medication, and it was shown to be associated with poor prognosis in CRC [15,16]. Other LncRNAs such as PVT-1 and MALAT1 were also related with CRC [17,18]. However, the overall pathophysiological contributions of LncRNAs to CRC remain largely unknown.

In the present study, we gained LncRNAs related with CRC by bioinformatics analysis, which is up-regulated in CRC compared with paired peritumoral tissues and several CRC cell lines. The effects of LncRNA DQ786243 were assessed by silencing it *in vitro* and *in vivo*.

## MATERIALS AND METHODS

### Cell culture and tissue specimens

All specimens were handled and made anonymous according to the ethical and legal standards. Paired tissue specimens (tumour and adjacent normal tissues) from 81 patients with CRC were obtained and histologically confirmed by a pathologist at Renji Hospital, Shanghai Jiao Tong University, from January 2010 to December 2012. Twenty of them were used to figure out LncRNAs aberrantly expressed in CRC. No patient has received preoperative treatment including chemotherapy, radiotherapy or any other adjuvant treatment. Resected tissue samples were immediately frozen in liquid nitrogen and stored at −80°C until RNA extraction. This study was approved by the institutional ethics committee of Shanghai Jiao Tong university, and written informed consent was obtained from each patient.

The human CRC cell lines, including SW620, HCT116 and HT29 were obtained from the A.T.C.C. All cell lines were maintained routinely in Dulbecco's modified Eagle's medium supplemented with 10% FBS and 2 mM L-glutamine (Invitrogen) and were grown at 37°C in a 10% CO_2_ atmosphere.

### Choice of differentially expressed LncRNAs list using heat map analysis

We obtained the microarray date from Gene Expression Omnibus (GEO, http://www.ncbi.nlm.nih.gov/geo/), and the GEO accession number is GSE3325. The date was generated using the genechip Affymetrix Human Genome U133 Plus 2.0 Array GPL570 (HG-U133_Plus_2), which completely coverage Human Genome U133 Set plus 6500 additional genes for analysis of over 47000 transcripts.

Observations with adjusted *P* values≥0.05 were removed, and thus excluded from further analysis. The heat map of the 50 LncRNAs most obvious differences was created using a method of hierarchical clustering by GeneSpring GX, version 7.3 (Agilent Technologies).

Chosen LncRNAs were finally confirmed for altered transcription level using quantitative real-time PCR (qRT-PCR) between tumour and adjacent normal tissues. Primers used in qRT-PCR were as follows: LncRNA DQ786243: 5′-agaggtgggagatgaggg-3′ (forward probe), 5′-cttctggcagcagtatgg-3′ (reverse probe). Other LncRNAs primer sequences are available upon request.

### RNA preparation, reverse transcription and quantitative real-time PCR

Total RNAs were extracted from tumorous and adjacent normal tissues using Trizol (Invitrogen) following the manufacturer's protocol. RT and qPCR kits were used to evaluate expression of LncRNA from tissue samples. The 20 μl of RT reactions were performed using a PrimeScript® RT reagent Kit (Takara) and incubated for 30 min at 37°C, 5 s at 85°C and then maintained at 4°C. For RT-PCR, 1 μl of diluted RT products were mixed with 10 μl of 2 × SYBR® PremixEx Taq™ (Takara), 0.6 μl forward and reverse primers (10 μM) and 8.4 μ of Nuclease-free water in a final volume of 20 μl according to manufacturer instructions. All reactions were run on the Eppendorf Mastercycler EP Gradient S (Eppendorf) using the following conditions: 95°C for 30 s, followed by 40 cycles at 95°C for 5 s and 60°C for 30 s. RT-PCR was done in triplicate, including no-template controls. Amplification of the appropriate product was confirmed by melting curve analysis following amplification. Relative expressions of LncRNAs were calculated using the comparative cycle threshold (*C*_T_; 2^−ΔΔCT^) method with glyceraldehyde-3-phosphate dehydrogenase (GAPDH) as the endogenous control to normalize the data.

### siRNA

Cells were seeded (2×10^5^ cells / well) in six-well plates. After incubation for 24 h, cells were transfected with siRNA targeting LncRNA or negative control (si-Scramble) using Lipofectamine 2000 transfection reagent. The sequences of siRNAs were as follows: si-DQ786243-1, 5′’-gccatgggtacccggatgatgttat-3′; si-DQ786243-2, 5′-ccatgggtacccggatgatgttata-3′; si-DQ786243-3, 5′-catgggtacccggatgatgttatat-3′; si-Scramble, 5′-gccgggcatgcctagtagtgattat-3′.

### Cell proliferation assay and cell cycle analysis

Cells were seeded in 96-well plates at 0.8–1×10^3^ per well. Cell proliferation was evaluated using Cell Counting Kit-8 (CCK-8; Beyotime) according to the manufacturer's instructions. Briefly, 10 μl of CCK-8 solution was added to culture medium, and incubated for 2 h. The absorbance at 450 nm wavelength was determined with a reference wavelength of 570 nm. For cell cycle analysis, cells were plated in six-well plates at 5×10^5^ per well. The cell-cycle distribution was analysed by propidium iodide (PI) (Sigma–Aldrich) staining and flow cytometry (FCM). All experiments were performed in triplicates.

### Apoptosis assay

Apoptosis was detected by FCM using Annexin V-FITC and PI apoptosis detection kit (Becton Dickinson). Briefly, adherent cells were harvested and suspended in the Annexin-binding buffer (1×10^6^ cells/ml). Thereafter, cells were incubated with Annexin V-FITC and PI for 15 min at room temperature in the dark and immediately analysed by FCM.

### Invasion assay

For invasion assays, matrigel-coated chambers (BD Biosciences) containing 8 μm pores were used for the assays. Briefly, 2×10^5^ cells were seeded into the upper chambers (coated in Matrigel) in serum-free medium. The lower chamber of the transwell was filled with culture media containing 10% FBS as a chemo-attractant. After the chambers were incubated at 37°C for 48 h, non-invaded cells on the top of the transwell were scraped off with a cotton swab. Cells, successfully translocated, were fixed with 10% formalin, stained with 0.1% crystal violet and counted under a light microscope.

### Wound healing assay

Cells were cultured in standard conditions until 80–90% confluence and treated with mitomycin C (10 μg/ml) during the wound healing assay. The cell migration was assessed by measuring the movement of cells into the acellular area created by a sterile insert. The wound closure was observed after 48 h.

### Western blot analysis

Cells were washed twice with cold PBS and lysed in radio-immunoprecipitation assay (RIPA) buffer (1×PBS, 1% NP40, 0.1% SDS, 5 mM EDTA, 0.5% sodium deoxycholate and 1 mM sodium orthovanadate) containing protease inhibitors. Whole protein extracts were resolved on a SDS/10% polyacrylamide gel and electrotransferred to polyvinylidene fluoride membranes (Millipore), which were then blocked in 5% non-fat dry milk in TBS (pH 7.5; 100 mM NaCl, 50 mM Tris and 0.1% Tween-20) and immunoblotted with specific primary antibodies against Caspase-3 (1:1000), Caspase-9 (1:1000), Bax (1:1500), Bcl-2 (1:1000), Cyclin A2 (1:2000), Cyclin B1 (1:1000), Cyclin D1 (1:5000), Cyclin E1 (1:1500), CDK4 (1:2000) and CDK6 (1:1000) (Santa Cruz Biotechnology) at 4°C overnight followed by HRP (horseradish peroxidase)-labelled secondary antibody (1:1000) (Santa Cruz Biotechnology) and detected by chemiluminescence. β-Actin expression was used as a protein-loading control. The intensity of protein bands was quantified with the Quantity One software (4.5.0 basic, Bio-Rad Laboratories).

### *In vivo* xenograft experiments

All BALB/c nude mice aged 6–7 weeks and weighing 20–22 g were used in the experiment. The animal study was performed at the Tongji University with approval from the Institutional Animal Care and Use Committee in accordance with the institutional guidelines. The BALB/c nude mice were administered with approximately 1×10^7^ cells in the log phase. Each experimental group consisted of four mice. After 100 days, the mice were killed and their tumours were excised [13,14]. The tumour weight was measured and the tumour volume was calculated according to the formula: Tumour volume (mm^3^)=(*wh*^2^)/2, where *w* is the longest axis (mm) and *h* is the shortest axis (mm).

### Statistical analysis

Data are reported as mean±S.D. Statistical significance was determined using double-sided Student's *t* test. Multiple groups were analysed using ANOVA. A *P* value of less than 0.05 was considered to be significant.

## RESULTS

### Differentially expressed LncRNAs between CRC tissues and adjacent non-cancer tissues

Hierarchical clustering showed systematic variations in the expression of LncRNAs between CRC and paired non-tumour samples (Figure 1A). To validate the microarray analysis findings, we selected ten LncRNAs among the differential LncRNAs and analysed their expression using qRT-PCR in 20 pairs of CRC and corresponding non-tumour tissues (Figure 1B). These data confirmed that AK026418, AK127644, AK095500, AK001058 and DQ786243 were overexpressed in CRC, whereas the expression of AK313307, AK026659, DQ679794, BC043558 and BC008657 were decreased. Thus, our data indicate that a set of LncRNAs is frequently aberrantly expressed in CRC tissues. It is also interesting that the expression of DQ786243 exhibits the greatest alteration in both CRC tissues and CRC cell lines (*P*<0.01; Figures 1C and 1D).

**Figure 1:** Differential expression of LncRNAs in CRC (**A**) Heat map analysis of the LncRNAs expression of groups was created using a method of hierarchical clustering by GeneSpring GX, version 7.3. Rows: samples; columns: LncRNAs; colour key indicates LncRNA expression value, red: highest, green: lowest. Microarray data were obtained from GEO, GSE number is GSE3325. (**B**) We validated the differential expression of six LncRNAs in three paired CRC and non-tumour samples using RT-PCR. (**C**) RT-PCR analysis of LncRNA DQ786243 expression in 20 paired CRC/non-tumour tissue specimens. (**D**) mRNA levels of LncRNA DQ786243 was detected by RT-PCR in CRC cell lines SW620, HCT116 and HT29. Data in histograms are means±S.D., *P<0.05, **P<0.01 compared with control cells (*t* test).

Together, these data indicate that abnormal DQ786243 expression may be related to CRC progression.

### Effect of LncRNA DQ786243 on CRC cell proliferation and apoptosis *in vitro*

As LncRNA DQ786243 expression level is significantly up-regulated in the tumour tissues of CRC, it may function as a tumour oncogene. To this end, we investigated whether knockdown of DQ786243 could suppress cell proliferation. As shown in Figure 1(D), among SW620, HCT116 and HT29 cells, the highest level of DQ786243 mRNA was found in SW620 cells, followed by HT29 cells. Thus, we silenced the expression of DQ786243 in SW620 and HT29 cells to examine the effects of DQ786243 on cell proliferation. Then, we transfected two siRNAs (LncRNA si-DQ786243 and si-Scramble) to silence the expression of DQ786243. CCK-8 assay showed that the silencing of DQ786243 notably retarded the cell proliferation in both SW620 and HT29 cells (*P*<0.01; Figure 2A).

**Figure 2:** Knockdown LncRNA DQ786243 inhibited cell proliferation and promoted cell apoptosis in SW620 and HT29 cells (**A**) CCK-8 assays were performed. DQ786243 silencing notably inhibited the cell proliferation in both SW620 and HT29 cells. The data represent the means±S.D. from three independent experiments. The error bars denote the S.D., **P<0.01. (**B**) Apoptosis was assessed using FCM. Representative quadrant figures were presented. Knockdown of DQ786243 greatly increased the number of total apoptotic cells in both SW620 and HT29 cells. (**C**) Immunoblotting assays were performed to examine certain apoptosis-related proteins in SW620 and HT29 cells transfected with si-DQ786243 or si-Scramble. β-Actin was used as an internal control. All the results shown are representative of three independent experiments, **P<0.01.

To determine whether apoptosis contributes to cell growth inhibition by LncRNA DQ786243 knockdown, we evaluated the effect of DQ786243 expression on cell apoptosis. Knockdown of DQ786243 greatly increased the number of total apoptotic cells in both SW620 and HT29 cells, indicating that the overexpression of DQ786243 may inhibit apoptosis in CRC cells (Figure 2B). To further study, possible mechanisms through which DQ786243 alters CRC cell proliferation, we examined the expression of certain genes involved in apoptosis regulation. As shown in Figure 2(C), DQ786243 knockdown in SW620 and HT29 cells decreased the expression of the anti-apoptotic protein Bcl-2, increased the expression of the pro-apoptotic proteins caspase-9 and caspase-3 and Bax.

These results suggest that the dysregulation of certain cell apoptosis-related proteins explains the DQ786243 dependent effects on CRC cell proliferation.

### LncRNA DQ786243 is involved in cell cycle progression

Because the induction of cell cycle arrest is an important anti-proliferation mechanism, we investigated whether the growth inhibitory activity of DQ786243 knockdown involved the control of cell cycle progression. As shown in Figure 3(A), the cell cycle progression of SW620 and HT29 cells were arrested at the G_2_/M-phase, whereas there were no significant differences in the cell-cycle distribution of the si-Scramble transfected cells and Blank. To examine the expression of intracellular proteins regulating cell cycle progression at G_2_/M-phase, we examined the level of Cyclin B1, CDC2 and p-CDC2. As shown in Figure 3(B), DQ786243 knockdown in SW620 and HT29 cells decreased the expression of Cyclin B1, CDC2 and *p*-CDC2. These data suggest that reduced CDC2-Cyclin B1 activity by knockdown of LncRNA DQ786243 is responsible for the G_2_/M arrest in our cell model system.

**Figure 3:** LncRNA DQ786243 regulated cell cycle progression in SW620 and HT29 cells (**A**) A cell cycle analysis was performed using FCM. Representative histograms were presented. Depletion of DQ786243 decreased the percentage of cells in S-phase and increased that in G_2_/M- phase in both SW620 and HT29 cells. All the results shown are representative of three independent experiments, **P<0.01. (**B**) Immunoblotting assays were performed to examine certain cell cycle-related proteins in SW620 and HT29 cells transfected with si-DQ786243 or si-Scramble.

These results suggest that the dysregulation of certain cell cycle-related proteins explains the DQ786243-dependent effects on CRC cell proliferation.

### Knockdown of LncRNA DQ786243 inhibits CRC migration and invasion

To determine whether LncRNA DQ786243 expression affected CRC migration and invasion, we performed wound healing and matrigel invasion assay using SW620 and HT29 cells. As shown in Figures 4(A) and 4(B), knockdown of LncRNA DQ786243 significantly suppressed cell migration and invasion (*P*<0.05). Previous studies have established that epithelial-mesenchymal transition (EMT) is required for metastasis in multiple human epithelium cancers [19,20]. Consequently, we measured EMT markers by western blot to evaluate whether DQ786243 could promote EMT-mediated CRC invasion. As shown in Figure 4(C), knockdown of DQ786243 suppressed E-cadherin expression, but increased expression of Vimentin and N-cadherin, compared with that in control cells (*P*<0.05). Moreover, notable transcription factors like ZEB1 expression was significantly inhibited in SW620 and HT29 cells. These results suggested that the reduced expression of LncRNA DQ786243 could weaken the invasion capacity and migration of CRC cells.

**Figure 4:** Knockdown LncRNA DQ786243 inhibited cell migration and invasion *in vitro* (**A**) Cell migratory abilities were measured by a wound healing assay. The wound areas were measured by ImageJ software. These data are shown as the mean±S.D. of three independent experiments. (**B**) Transwell invasion (crystal violet staining, original magnification ×200). SW620 and HT29 cells transfected with si-DQ786243 had a little cells migrated through the basement membrane, compared with si-Scramble and Blank groups (**P<0.01). No significant difference was observed between si-Scramble group and Blank group (*P* > 0.05). (**C**) The expression of EMT-related proteins in SW620 and HT29 cells by western blot. The levels of ZEB1 and E-cadherin were down-regulated in SW620 and HT29 cells transfected with si-DQ786243 (*P<0.05, **P < 0.01). But, the expression of Vimentin and N-cadherin were significantly increased in the both cells (**P<0.01).

### Knockdown of LncRNA DQ786243 suppressed tumorigenicity of CRC cells *in vivo*

To further verify the role of DQ786243 and to determine the therapeutic potential of targeting DQ786243 in CRC, we established xenograft tumour models using SW620 and HT29 cells. The tumour weight and tumour growth curve suggested that DQ786243 inhibition suppressed effectively tumour growth comparing with the scramble treated xenograft tumours (*P*<0.05, Figures 5A and 5B). These results suggest that down-regulating DQ786243 inhibits tumour growth *in vivo*.

**Figure 5:** Knockdown LncRNA DQ786243 inhibited the growth of CRC cells *in vivo* Nude mice were injected with SW620 and HT29 cells transfected with si-DQ786243 or si-Scramble via the peritoneal injection. After 14 weeks, mice were killed and tissues were harvested for analysis. (**A**) Knockdown of LncRNA DQ786243 in CRC cells significantly inhibits tumour growth in a mouse xenograft model; *P<0.05, **P<0.01 compared with si-Scramble. (**B**) Tumour weights of corresponding mouse xenograft models; *P<0.05, **P<0.01 compared with si-Scramble.

## DISCUSSION

Emerging evidence indicates LncRNAs play a pivotal role in several cancers [21–24]. In the present study, we have identified a small number of LncRNAs that are aberrantly expressed in human CRC compared with paired peritumoral tissues. Our functional assays revealed that DQ786243 suppression decreased cell proliferation both *in vitro* and *in vivo*. Furthermore, we found that silencing DQ786243 retarded cell cycle progression, promoted cell apoptosis and inhibited CRC migration and invasion in SW620 and HT29 CRC cells. These findings suggest DQ786243 may be an oncogene that promotes CRC progression.

It has been previously demonstrated that protein-coding genes account for only 2% of the total genome, whereas the vast majority of the human genome can be transcripted into non-coding RNAs [25]. Among these, LncRNAs have been certified as important biological RNAs in the post-transcriptional regulation of the target genes [26]. For example, MALAT-1 has been reported to promote cell migration/invasion in lung cancer and oral squamous cell carcinoma, and HULC has been implicated in the regulation of hepatoma cancer cell proliferation [27,28]. Enhanced expression of LncRNA ZXF1 also promoted the invasion and metastasis in lung adenocarcinoma [29]. Furthermore, the H19, MEG3 and BC200 were deregulated in many kinds of cancer [10,30–32]. Despite these findings, the overall pathophysiological contributions of LncRNAs to CRC remain largely unknown.

In the present study, we identified LncRNA DQ786243 as a differentially between CRC tissues and paired adjacent normal tissues. Our functional assays revealed that DQ786243 suppression decreased cell proliferation both *in vitro* and *in vivo*, indicating that it plays a crucial role in promoting CRC proliferation. To investigate the possible mechanism responsible for the proliferation enhancement effect of DQ786243, we performed FCM assay and found that silencing DQ786243 arrested cell cycle at G_2_/M-phase, promoted cell apoptosis and inhibited CRC migration and invasion in SW620 and HT29 CRC cells, indicating that DQ786243-mediated CRC cell proliferation may be associated with the regulation of the cell cycle and apoptosis. To further elucidate the regulatory mechanism of DQ786243 in cell cycle and apoptosis, proteins involved in cell cycle and apoptosis were analysed by immunoblotting. Our results indicated that silencing DQ786243 markedly decreased the expression of Cyclin B1 and the phosphorylated level of CDC2. It has been widely accepted that Cyclin B1–CDC2 complex is required for cells transition from G_2_ to M-phase [29]. We also observed that DQ786243 knockdown in SW620 and HT29 cells decreased the expression of the anti-apoptotic protein Bcl-2, increased the expression of the pro-apoptotic proteins caspase-9, caspase-3 and Bax. These results may extend our current knowledge about the downstream genes of DQ786243 to include these cell cycle- and apoptotic-related proteins.

Interestingly, our data also showed that the knockdown of DQ786243 in SW620 and HT29 cells resulted in an increase in N-cadherin and Vimentin protein levels but a decrease in the ZEB1 and E-cadherin protein level, indicating LncRNA DQ786243 regulated EMT process via classical signal pathways.

Though some LncRNAs have reported involving in the progression and development of tumours, the underlying molecular mechanism is still unclearly elucidated. In the present study, we found that LncRNA DQ786243 expressions were related in CRC cell lines. Of course, as the number of available CRC cell lines was limited and these cultured cell lines cannot stand for all subtypes of colorectal tumour, a more systemic study using clinical CRC samples is required, however, it provided a possibility that the overexpression of LncRNA DQ786243 may be involved in colorectal tumorigenesis.

In summary, the present study has shown that LncRNA DQ786243 expression is up-regulated in CRC tissues and cells. We have shown that LncRNA DQ786243 can regulate cancer cell proliferation, cell cycle progression, cell apoptosis migration and invasion. Taken together, these findings contribute to a better understanding of the importance of dysregulated LncRNAs in CRC progression and provide a rationale for the potential development of LncRNA-based targeted approaches for the treatment of CRC.

## Abbreviations

CCK-8: Cell Counting Kit-8
CRC: colorectal cancer
EMT: epithelial-mesenchymal transition
FCM: flow cytometry
GEO: Gene Expression Omnibus
LncRNA: long non-coding RNA
PI: propidium iodide
RIPA: radio-immunoprecipitation assay
